RETRACTED

# Dehydroevodiamine suppresses inflammatory responses in adjuvant-induced arthritis rats and human fibroblast-like synoviocytes

**DOI:** 10.1080/21655979.2021.1999554

**Published:** 2021-12-27

**Authors:** Yufang Dai, Jiaoe Sheng, Sanshan He, Qingchao Wu, Yunlong Wang, Linchong Su

**Affiliations:** Department of Rheumatology and Immunology, Minda Hospital of Hubei Minzu University, Hubei Provincial Key Laboratory of Occurrence and Intervention of Rheumatic Disease, Enshi, China

**Keywords:** Dehydroevodiamine, rheumatoid arthritis, aia, mh7a, mapk

## Abstract

Dehydroevodiamine (DHE) is an effective natural active substance extracted from *Euodiae Fructus*, which is a widely used herbal drug in traditional Chinese medicine. The focus of this study was to test the possibility of using DHE in the treatment of rheumatoid arthritis (RA) diseases. A rat model of adjuvant-induced arthritis (AIA) was generated using Complete Freund’s Adjuvant (CFA). Body weight changes, arthritis scores, ankle pathology, tumor necrosis factor-alpha (TNF-α), interleukin-1β(IL-1β), interleukin-6 (IL-6), and interleukin-17 (IL-17) secretion, as well as matrix metalloproteinase (MMP) expression in joint tissue, were measured as indicators of viability of DHE medicated AIA rats. Human fibroblast-like synoviocytes (MH7A cells) were connected to check these impacts. The results confirmed that DHE administration had an excellent therapeutic impact on the AIA rat model, substantially relieving joint swelling, inhibiting synovial pannus hyperplasia, and decreasing joint scores. In addition, the serum enzyme-linked immunosorbent assay (ELISA) showed that DHE treatment reduced the expression of pro-inflammatory factors in AIA rats. The immunohistochemical results showed that DHE treatment could reduce the synthesis of MMPs such as matrix metalloproteinase-1(MMP-1) and matrix metalloproteinase-3 (MMP-3) in the ankle tissue of AIA rats. In vitro, DHE inhibited cell proliferation, mRNA transcription, protein synthesis of proinflammatory factors such as IL-1βand IL-6, and matrix metalloproteinases such as MMP-1 and MMP-3. Furthermore, DHE inhibited the phosphorylation levels of p38, JNK, and ERK proteins in TNF-α-treated MH7A cells.This work assessed the effect of DHE in AIA rats and revealed its mechanism in vitro.

## Introduction

Rheumatoid arthritis (RA) is an intractable immune disorder with clinical symptoms of joint deformity and redness, and its onset may be associated with genetic and environmental factors [1]. In the RA process, the synovium is transformed into proliferative invasive tissue, causing cartilage and bone damage. Fibroblast-like synoviocytes (FLSs) are mesenchymal cells in the synovium of the joint, which produce inflammatory factors, synthesize metal matrix enzymes, and are critical for the development of RA [2].

RETRACTED

The current treatment strategy is aimed at the end-stage of the disease and is broadly anti-inflammatory. Recognizing that RA goes through a relatively stable stage and the molecular characteristics of the relevant transition points, it is possible to identify the upstream targets, to prevent the disease process before irreversible tissue damage occurs [3]. Seeking effective drug treatment for RA has attracted increased attention. Many small molecules extracted from natural products such as Chinese herbal medicines can improve the outcome of RA treatment by reducing inflammation and inhibiting the abnormal proliferation of fibroblasts. For example, Astragalin ameliorated bone damage and joint inflammation in a collagen-induced arthritis (CIA) mouse model by inhibiting the production of MMPs in fibroblasts by regulating the mitogen-activated protein kinase (MAPK)/AP-1 pathway [4]. Network pharmacology studies have shown that Compound Fengshiding capsules treat RA through anti-apoptotic, anti-inflammatory, and antioxidant stress effects [5]. Salicin improves RA, which may be related to oxidative stress and the Nrf2-HO-1-ROS pathway in RA-FLSs [6].

*Euodiae Fructus* is a Chinese herbal medicine commonly used in Chinese folk for its analgesic efficacy, and dehydroevodiamine (DHE) is a natural small molecule product derived from *Euodiae Fructus* [7]. DHE has been shown to have good pharmacological activity, such as neuroprotective and cardiovascular protective effects [8,9]. DHE has been reported to show better anti-inflammatory effects in *in vitro* cell models, such as its ability to inhibit nuclear factor-kappaB (NF-κB) pathway in lipopolysaccharide (LPS)-stimulated macrophages [10]. However, there are no reports on its treatment for RA. Therefore, the purpose of our study was to explore the therapeutic effect of DHE on RA in CFA-induced AIA model rats and initially explore the potential mechanism of the effect of DHE on RA induced in FLS-MH7A cells.

## Materials and methods

### Drugs and reagents

Dehydroevodiamine (purity > 99%) was purchased from the Southwest Standards R&D Center (Chengdu, China). Methotrexate (MTX) was procured from Shanghai Xinyi Pharmaceutical Factory Co., Ltd. (Shanghai, China). Complete Freund’s Adjuvant (CFA, #7027) was purchased from Chondrex (Redmond, WA, USA).

### Animal model establishment and administration

Sprague-Dawley (SD) rats weighing 100–120 g were purchased from the Laboratory Animal Center for Medical Sciences, Three GORGES University (SCXK (Hubei, China) 2015–0018). Throughout the experiment, the rats were housed in a temperature and humidity-appropriate specific-pathogen-free animal house, given adequate diet and water, daily light for 12 h, and adaptively housed for a week before starting the experiment. At the same time, the welfare and treatment of the animals were fully secured in compliance with the rules and regulations of the Animal Care and Use Committee at Minda Hospital of Hubei Minzu University.

RETRACTED

First, after 7 days of adaptive feeding, we randomly divided 40 rats into 5 groups: normal group (Con), model group (Mod), positive drug group (MTX), DHE low-dose group (DHE 10 mg/kg), and DHE high-dose group (DHE 20 mg/kg). Except for the normal group, 0.1 ml of CFA (10 mg/ml) was injected subcutaneously at the root of the tail for modeling [11]. In the animal experiments, we used 0.5% carboxyl methyl cellulose (CMC)-Na to dissolve the DHE. From the first day after modeling, the groups were dosed separately starting with drug administration as outlined in the flow chart in Figure 1b.

**Figure 1.** (a) Molecular structure of dehydroevodiamine (DHE). (b) Flow chart of animal experiment modeling and administration. Control (Con), model (Mod), dehydroevodiamine (DHE), methotrexate (MTX), Complete Freund’s Adjuvant (CFA).

### Criteria for joint scoring

The adjuvant arthritis rat models were considered successful when at least one finger or paw was swollen. The arthritis scoring criteria was: 0 – normal, no swelling; 1 – slight swelling of skin and swelling of joints; 2 – moderate or mild swelling of feet, pads, or ankles; 3 – severe and moderate swelling of feet, toes, and joints; and 4 – severely and highly swollen feet, toes, and joints, without stiffness or deformity [12].

### Histopathological assessment

The decalcified wax blocks were sectioned, then fixed in 95% ethanol for 20 min, washed with phosphate-buffered saline (PBS) twice for 1 min, and stained with hematoxylin solution for 2–3 min to dye the nuclei. Then, the tissue was washed with tap water, and observed under the microscope. Next, the tissue was immersed in eosin solution for 1 min to dye the cytoplasm. After washing with tap water, the tissue was blown dry or allowed to dry naturally, and cover-slipped and sealed with a neutral gum [13].

### Immunohistochemical analysis

Paraffin-embedded ankle tissue was sectioned and rinsed with PBS after dewaxing. After deparaffinization and the removal of catalase by adding 3% H_2_O_2_, the antigen sites were exposed by steaming twice after washing. After antigen retrieval, blocking was performed with serum. After blocking was completed, MMP-1 (Abcam, # ab52631) and MMP-3(Abcam, # ab52915) antibodies were added at 4°C overnight. After removal, the tissue was washed in PBS, followed by incubation with the secondary antibody. After washing in PBS, the color reagent was added. Finally, the specimens were observed and photographed under a microscope [14].

RETRACTED

### Fibroblast sources and culture

The RA-FLSs (MH7A) cell line was purchased from the Beijing Beina Biology Co., Ltd (Beijing, China). The MH7A cell line was cultured in 1640 medium (Gibco, California, USA), incubated in 5% CO_2_ at 37°C, subcultured every 3–5 days, and digested with trypsin without ethylenediaminetetraacetic acid (EDTA) [15].

### Cell proliferation

MH7A cells were cultured at a density of 5000 cells per well in 96-well plates for 24 hours and divided into 5 groups. Except for the blank cell group, the other 4 groups were treated with 10 ng/ ml TNF – α for 24 h. Three groups were treated with DHE at concentrations of 5 μM,10 μM, and 20 μM. Medium with 0.1% dimethylsulfoxide (DMSO) was used to treat the control group cells. In the cell experiments, DMSO was used to dissolve DHE. After 24 h, 10 uL of CCK-8 reagent was added to each well and incubated for 2 h. The absorbance of each well was measured at a wavelength of 450 nm [16].

### Determination of inflammatory factors

The serum of DHE-treated AIA rats was collected using blood collection tubes, centrifuged at 3000 rpm for 15 min, and the supernatant was collected. The protein levels of TNF-α (Elabscience, # E-EL-R0019c, WuHan, China), IL-1β, IL-6, and IL-17 (Elabscience, # E-EL-R0566c, WuHan, China) were measured according to the ELISA kit instructions. MH7A cells were seeded at a density of 5 × 10^5^ cells per well on 12-well plates for 24 hours and divided into 5 groups. Except for the blank cell group, the other 4 groups were treated with 10 ng/ml TNF – α for 24 h. Three groups were treated with DHE at concentrations of 5 μM, 10 μM, and 20 μM, and the control group received medium containing 0.1% DMSO. After incubating for 24 hours, the cell supernatant was removed and IL-6 (Elabscience, # E-EL-R0896c) and IL-1β (Elabsandcience, # E-EL-R0012c) were analyzed according to the ELISA kit instructions [17].

### Reverse-transcription PCR (RT-PCR)

MH7A cells seeded at a density of 1 × 10^6^ cells per well were cultured on 6-well plates for 24 hours and divided into 5 groups. Except for the blank cell group, the other 4 groups were treated with 10 ng/ mL TNF – α for 24 h. Three groups were treated with DHE at concentrations of 5 μM, 10 μM, and 20 μM and the control group cells received medium containing 0.1% DMSO. After incubation for 24 hours, total RNA was extracted using Trizol and the concentration and purity of the extracted RNA were detected, reverse transcribed into cDNA, and the relative IL-6, IL-1β, MMP1, and MMP3 contents were detected by RT-PCR [18]. The IL-6, IL-1β, MMP1, and MMP3 primers were designed by Shanghai Shenggong Biosynthesis. Detailed primer information is provided in Table 1.

RETRACTED

**Table 1.** Primers used in RT-PCR

Primer name	species	Primer sequence (5 ‘ – 3ʹ)
IL-1β (F)	Human	5ʹ-CTTCAGGCAGGCAGTATCACTC – 3ʹ
IL-1β (R)	Human	5ʹ-TGCAGTTGTCTAATGGGAACGT – 3ʹ
IL-6 (F)	Human	5ʹ-CCCCACCCTCACCCTCCAAC – 3ʹ
IL-6 (R)	Human	5ʹ-TGGGCTCGAGGGCAGAATGAG – 3ʹ
MMP-1(F)	Human	5ʹ-CTCAATTTCACTTCTGTTTTCTG – 3ʹ
MMP-1(R)	Human	5ʹ – CATCTCTGTCGGCAAATTCGT-3ʹ
MMP-3(F)	Human	5ʹ-GGCTTCAGTACCTTCCCAGG – 3ʹ
MMP-3(R)	Human	5ʹ-GCAGCAACC AGGAATAGGTT – 3ʹ
Actin(F)	Human	5ʹ-TGCTGTCCCTGTATGCCTCT – 3ʹ
Actin(R)	Human	5ʹ-TTTGATGTCACGCACGATTT – 3ʹ

### Western blotting

MH7A cells were seeded at a density of 10^6^ cells per well on 6-well plates for 24 hours and divided into 5 groups. Except for the blank cell group, the other 4 groups were treated with 10 ng/ mL TNF – α for 24 h. Three groups were treated with DHE at concentrations of 5 μM, 10 μM, and 20 μM. The control group received medium containing 0.1% DMSO. After incubating for 24 hours, the cells were rinsed three times in cold PBS, and protein was collected by adding protein lysis buffer containing protease inhibitors. The total proteins were separated by sodium dodecyl sulfate-polyacrylamide gel electrophoresis, followed by wet blotting, blocking with milk after membrane shift, and incubating with antibodies against P-P38 (CST,#4511), MMP-1 (Abcam,# ab134184), MMP-3 (Abcam,# ab52915), SAPK/JNK (CST,#9252), P44/42 MAPK (ERK 1/2) (CST,#4695), P-P44/42 MAPK (T202/Y204) (CST,#4370), P38 (CST,#8690), and P-SAPK/JNK (T183/Y185) (CST,#9255) at 4°C overnight. After removal, they were rinsed and then incubated with the secondary antibody, and finally color development was performed and photographed by an imaging system [19].

### Statistical analysis

GraphPad Prism software (version 5.0) was used for all data analyses in this study. The data are indicated as means ± SEM. We employed the Student’s t-test to analyze the variations between two groups, and one-way ANOVA with Bonferroni’s correction to assess more than two groups. P < 0.05 indicated significant difference.

## Results

### DHE inhibits disease progression in AIA rats

To characterize the anti-arthritis efficacy of DHE, a CFA-induced AIA rat model was used to evaluate the therapeutic effect of RA. From the 12th day after CFA injection, except for the normal group, the ankles, toes, and whole legs of rats in the other groups had varying degrees of redness and swelling. After 30 days of treatment, the ankle swelling in the untreated model group was the most serious, whereas the swelling in the high-dose DHE group was the least, followed by the positive drug group, and the ankles in the mice in the low-dose DHE group were swollen as well (Figure 2a). Considering that weight loss is the principal medical characteristic of RA, we investigated the weight of AIA rats in each treatment group for 30 days. Compared to the control group, the weight of rats in each group treated with tail root injection of CFA increased slowly. Among them, the weight increase in the rats in the Mod group was the slowest, and significantly different from the normal group on the 30th day (p < 0.05). Treatment with different DHE concentrations and MTX significantly inhibited the weight loss of AIA rats compared to the Mod group (p < 0.05), with the best efficacy in the high-dose DHE group (Figure 2b). Additionally, the joint scores of the AIA rats were increased from day 12 after CFA injection and reduced in all treatment groups. Compared to the MTX group, the high-dose DHE group exhibited a more pronounced effect (Figure 2c).

RETRACTED

**Figure 2.** (a) Visual diagram of rat foot swelling in each group on the 30th day after CFA injection. (b) Body weight changes in rats in each group at 30 days. (c) Arthritis scores of rats 30 days after the administration of dehydroevodiamine (DHE), Control (Con), model (Mod), dehydroevodiamine (DHE), methotrexate (MTX). The data are presented as the mean values of replicates ± SEM using one-way ANOVA with t-test, n = 8. ^#^p < 0.05, ^##^p < 0.01 compared to the control group, **p < 0.01, and *p < 0.05 compared to the model group.

## DHE inhibits ankle lesions in AIA rats

After decalcification of the ankle joints, hematoxylin and eosin (H&E)-stained sagittal sections showed that after AIA modeling, ankle joint swelling led to obvious stenosis of the joint cavity, accompanied by cartilage matrix injury. Both the DHE high-dose group and the MTX group showed significant inhibition of cartilage matrix injury and joint cavity stenosis (Figure 3).

**Figure 3.** H&E staining of sagittal sections after the decalcification of ankle joints of rats in each group (100**× **magnification). Control (Con), model (Mod), dehydroevodiamine (DHE), methotrexate (MTX).

## DHE inhibits the secretion of pro-inflammatory factors in the serum of AIA rats

After CFA injection, the serum pro-inflammatory factors such as TNF – α, IL-6, IL-1 β, and IL-17 were increased significantly. After 30 days of treatment, the different DHE doses and MTX effectively inhibited the abnormal increase in pro-inflammatory factors in AIA rats. The inhibition was greatest in the high-dose DHE group (Figure 4a-d).

RETRACTED

**Figure 4.** ELISA kits were used to measure proinflammatory factors in the serum of rats in each group. (a) TNF-α, (b) IL-1β, (c) IL-6, (d) IL-17. Dehydroevodiamine (DHE), methotrexate (MTX). The data are presented as the mean values of replicates ± SEM using one-way ANOVA with t-test, n = 8. ^#^p < 0.05, ^##^p < 0.01 compared to the control group, **p < 0.01, and *p < 0.05 compared to the model group.

## DHE inhibits the expression of MMPs in AIA rats

Immunohistochemically stained sections showed that the positive expression of MMPs in the ankle tissues of AIA rats increased significantly after CFA injection. The expression of MMP-1 and MMP-3 expressed in the cartilage and synovium of AIA rats increased significantly but decreased after treatment with 20 mg/kg DHE (Figure 5).

**Figure 5.** The expression of MMP-1 (a) and MMP-3 (b) in the ankle tissues of the normal group, model group, and high-dose DHE group was observed by immunohistochemical staining (200**× **magnification).

## DHE inhibits the proliferation of TNF-a-induced MH7A Cells

Compared with no TNF-α induction, in the groups treated with TNF-α for 24 hours, the MH7A cells proliferated faster, while after treatment with different concentrations of DHE, the cell proliferation rate decreased in a dose-dependent manner (Figure 6a). Statistical analysis showed that DHE at concentrations of 5, 10, and 20 μM could significantly inhibit TNF – α-induced fibroblast proliferation (Figure 6b).

**Figure 6.** (a) MH7A cells were treated or untreated with 10 ng/ml TNF – α for 24 hours. At the same time as TNF-α induction, the cells were treated with 5, 10, and 20 μM DHE for 24 hours. The effect on cell proliferation was observed. (b) A CCK8 kit was used to detect the absorbance of cell proliferation for 24 hours. The data are presented as the mean values of replicates ± SEM using one-way ANOVA with t-test, n = 10. ^#^p < 0.05, ^##^p < 0.01 compared to the control group, **p < 0.01, and *p < 0.05 compared to the model group.

## DHE suppresses the expression of pro-inflammatory factors in TNF-a-induced MH7A cells

After 24 hours of TNF-α induction, the pro-inflammatory factors IL-6 and IL-1β in MH7A cell lysates and cell supernatants were measured by RT-PCR and ELISA. The mRNA and protein levels of IL-6 and IL-1β were significantly higher than in cells without TNF – α induction (p < 0.01). DHE treatment at 5 μM did not inhibit the increase in IL-6 and IL-1β, but 10 μM and 20 μM, DHE significantly reduced the increase in IL-6 and IL-1β (p < 0.01) (Figure 7a-d).

**Figure 7.** MH7A cells were treated or untreated with 10 ng/ml TNF – α for 24 hours. At the same time, the cells were treated with DHE at concentrations of 5, 10, and 20 μM for 24 hours. ELISA was used to measure the expression of pro-inflammatory factors IL-6 (a) and IL-1β (b) in the supernatant of MH7A cells after 24 hours. RT-PCR was used to detect the expression of pro-inflammatory factors IL-6 (c) and IL-1β (d) in the lysate of MH7A cells after 24 hours. The data are presented as the mean values of replicates ± SEM using one-way ANOVA with t-test, n = 8. ^#^p < 0.05, ^##^p < 0.01 compared to the control group, **p < 0.01, and *p < 0.05 compared to the model group.

RETRACTED

## DHE inhibits MMPs synthesis in MH7A cells

To verify the inhibitory effect of DHE on the synthesis of MMPs in fibroblast synovial cells, TNF – α MH7A cells were stimulated for 24 hours and treated with different concentrations of DHE. The results showed that after 24 hours of TNF – α stimulation, the mRNA and protein levels of MMP-1 and MMP-3 increased significantly, while 10 μM and 20 μM DHE significantly inhibited the mRNA and protein levels of MMP-1 and MMP-3 (Figure 8a-f).

**Figure 8.** MH7A cells were treated or untreated with 10 ng/ml TNF-α for 24 hours. At the same time, the cells were treated with DHE at concentrations of 5, 10, and 20 μM for 24 hours. RT-PCR was used to detect the expression of MMP-1 (a) and MMP-3 (b) in the lysate of MH7A cells after 24 hours. Western blotting was used to detect the expression of MMP-1 (c) and MMP-3 (e) in the lysate of MH7A cells after 24 hours. (d, f) The relative density of each signaling band was calculated. The data are presented as the mean values of replicates ± SEM using one-way ANOVA with t-test, n = 3. ^#^p < 0.05, ^##^p < 0.01 compared to the control group, **p < 0.01, and *p < 0.05 compared to the model group.

## DHE inhibits the expression of MMPs by regulating MAPK signaling pathway

The MAPK pathway proteins are closely related to the production of inflammatory factors and MMPs [20,21]. To further explore whether the mechanism of DHE in inhibiting the expression of MMPs was related to the activation of the MAPK signaling pathway, we used TNF – α to stimulate MH7A cells for 24 hours, and treated them with different concentrations of DHE. After collecting the proteins, Western blot analysis was performed. The results showed that, after TNF-α stimulation, the MAPK pathway was activated and the phosphorylation levels of p38, ERK, and JNK increased significantly, while treatment with 10 μM and 20 μM DHE significantly inhibited their phosphorylation levels (Figure 9a**–D)**.

**Figure 9.** MH7A cells were treated or untreated with 10 ng/ml TNF – α for 24 hours. At the same time, the cells were treated with DHE at concentrations of 5, 10, and 20 μM for 24 hours. (a) Western blotting was used to detect the expression of p-p38, p38, p-JNK, JNK, p-ERK, and ERK in the lysate of MH7A cells after 24 hours. **(B, C, D)** The relative density of each signaling band was calculated. The data are presented as the mean values of replicates ± SEM using one-way ANOVA with t-test, n = 3. ^#^p < 0.05, ^##^p < 0.01 compared to the control group, **p < 0.01, and *p < 0.05 compared to the model group.

RETRACTED

## Discussion

In this study, we first evaluated the efficacy of DHE in treating RA with the aid of an AIA animal model and further revealed the mechanism of action of DHE in treating RA through an *in vitro* induction model in human fibroblasts. Our study confirmed that DHE administration had an excellent therapeutic impact on the AIA rat model, substantially relieving joint swelling, inhibiting synovial pannus hyperplasia, and decreasing joint scores. *In vitro* cell experiments verified the efficacy of DHE in the treatment of RA, and preliminarily revealed that the effect was due to reducing inflammation and MMPs by regulating the MAPK pathway.

RA is a common and typical inflammatory disease that, if left untreated, will eventually lead to severe joint damage and seriously affect the patient’s quality of life. RA may increase the incidence of some diseases, such as associated interstitial lung disease and idiopathic pulmonary fibrosis [22]. Due to the influence of traditional and non-traditional risk factors, the risk of cardiovascular disease in patients with RA is higher than that in the general population [23]. Traditional drugs and biological agents for the treatment of RA have been proved to improve the clinical symptoms of patients. However, their side effects, high price, and drug tolerance cannot be ignored [24]. Therefore, finding more effective, low-cost drugs with fewer side effects from natural herbs, fruits, and other natural products has become important. In this study, we found that DHE showed a good therapeutic effect on RA in AIA model rats, and could significantly inhibit weight loss, joint swelling, and cartilage damage.

Fibroblasts are the main component of the inner wall of the joint cavity called the synovium. During joint inflammation, fibroblasts promote the recruitment and retention of inflammatory cells by producing inflammatory mediators at pathogenic levels, thereby contributing to disease pathology [25]. The MH7A synovial fibroblast cell line used in this experiment is a chemically treated cell line extracted from the synovium of a female RA patient using SV40 T antigen. The cell line can be stably propagated for 10–15 generations. In recent years, it has made the screening of RA drugs and the exploration of the mechanism of RA drug treatment more convenient [26]. TNF-α is a major inflammatory mediator in the pathogenesis of RA as it can promote RA symptoms such as the secretion of inflammatory cytokines; fibroblast proliferation, migration, and invasion; and the synthesis of MMPs, etc. Therefore, TNF-α is often used to treat fibroblasts *in vitro* to simulate RA [27]. Our study showed that DHE could significantly inhibit cell proliferation in TNF-α-stimulated fibroblasts.

RETRACTED

The most significant feature of RA is the inability to control the excessive release of inflammatory factors. Controlling inflammation can prevent the development of the disease, which is the best strategy for RA treatment [28]. Thus, more and more TNF monoclonal antibody drugs have been developed and applied in major hospitals worldwide to treat RA [29]. Many studies have shown that fibroblasts and macrophages secrete IL-6 during the pathogenesis of RA. IL-6 can activate the assembly of NLRP3 inflammatory bodies and promote macrophages to produce IL-1β[Wang, 30]. IL-17 is a cytokine produced by Th17 cells. A systematic analysis of multiple databases showed that IL-17 was significantly correlated with the susceptibility to and clinical symptoms of RA patients [31]. Our study showed that DHE could not only inhibit the expression of four pro-inflammatory factors in AIA rats but also inhibit TNF-α-stimulated MH7A cells to secrete pro-inflammatory factors such as IL-6 and IL-1β.

MMPs is a type of zinc-dependent endopeptidase, which is the main protease used to invade and degrade the basement membrane and extracellular matrix [32]. The MMP family has many subtypes, such as MMP-1, MMP-2, MMP-3, MMP-9, and MMP-13 [33]. Different MMPs play different roles in different diseases and stages, and different drugs will also affect different kinds of MMPs [34]. There are many reports on the abnormal increases in MMP-1, MMP-2, MMP-3, MMP-9, and MMP-13 in RA [35,36]. Our study showed that DHE could not only inhibit the expression of MMP-1 and MMP-3 in the ankle synovia of AIA model rats, but also inhibit the production of MMP-1 and MMP-3 by fibroblast synovial cells stimulated by TNF-α. Accumulating evidence has shown that the production of pro-inflammatory factors and MMPs were closely related to the MAPK signaling pathway [36]. Our study showed that DHE could regulate the phosphorylation of MAPK pathway proteins p38, ERK, and JNK. It is speculated that the anti-inflammatory and MMP-inhibiting effects of DHE may be related to the MAPK pathway.

In summary, our study reported the anti-RA effect of DHE for the first time, and that DHE was a potential anti-inflammatory drug. At the same time, the efficacy of DHE was verified in fibroblast synovial cells *in vitro* and its mechanism was discussed. However, our findings are preliminary, and the study had many limitations, which are worthy of addressing in the future. First, the immunological mechanism of DHE was not deeply investigated in this study. In the next step, we will explore the mechanism of DHE in the treatment of RA from an immunologic perspective. Secondly, the AIA rat model is only one type of RA model, which has some defects and deficiencies. We plan to use different kinds of animals in the next series of experiments to verify the efficacy of DHE. In addition, this study did not deeply explore the molecular mechanism of the drug’s action. We will continue to explore its mechanism from different angles.

RETRACTED

## Conclusions

In this project, we discussed whether DHE had a manageable protective effect on adjuvant-induced RA and mentioned its feasible mechanism. The CFA-induced AIA rat model and the TNF-α-induced MH7A fibroblast model were used to investigate the efficacy and reveal the mechanism of action on RA. Our study results showed that DHE could significantly improve the weight loss, joint redness, and joint swelling of AIA rats, and inhibit the production of systemic pro-inflammatory factors and MMPs in tissues. DHE was also found to inhibit cell proliferation in TNF-α-induced fibroblasts and inhibit the production of pro-inflammatory factors and MMPs, and its mechanism may be related to the regulation of the MAPK pathway.

## Supplementary Material

Supplemental Material

## Abbreviations

MMP-3, matrix metalloproteinases-3; DHE, Dehydroevodiamine; AIA, adjuvant-induced arthritis; RA, Rheumatoid arthritis; IL-6, interleukin-6; MTX, Methotrexate. TNF-α, Tumor necrosis factor-alpha; IL-1β, Interleukin-1β; MMP-1, matrix metalloproteinases-1; MAPK, mitogen-activated protein kinases; IL-17, interleukin-17; CFA, complete Freund’s adjuvant;LPS, Lipopolysaccharide.
